RETRACTED

# System Accuracy Evaluation of the GlucoRx Nexus Voice TD-4280 Blood Glucose Monitoring System

**DOI:** 10.1155/2014/602586

**Published:** 2014-10-13

**Authors:** Muhammad Khan, Keith Broadbent, Mike Morris, David Ewins, Franklin Joseph

**Affiliations:** ^1^Department of Diabetes & Endocrinology, Countess of Chester Hospital NHS Foundation Trust, Chester CH2 1UL, UK; ^2^Department of Clinical Sciences & Nutrition, University of Chester, Chester CH1 4BJ, UK

## Abstract

Use of blood glucose (BG) meters in the self-monitoring of blood glucose (SMBG) significantly lowers the risk of diabetic complications. With several BG meters now commercially available, the International Organization for Standardization (ISO) ensures that each BG meter conforms to a set degree of accuracy. Although adherence to ISO guidelines is a prerequisite for commercialization in Europe, several BG meters claim to meet the ISO guidelines yet fail to do so on internal validation. We conducted a study to determine whether the accuracy of the GlucoRx Nexus TD-4280 meter, utilized by our department for its cost-effectiveness, complied with ISO guidelines. 105 patients requiring laboratory blood glucose analysis were randomly selected and reference measurements were determined by the UniCel DxC 800 clinical system. Overall the BG meter failed to adhere to the ≥95% accuracy criterion required by both the 15197:2003 (overall accuracy 92.4%) and 15197:2013 protocol (overall accuracy 86.7%). Inaccurate meters have an inherent risk of over- and/or underestimating the true BG concentration, thereby risking patients to incorrect therapeutic interventions. Our study demonstrates the importance of internally validating the accuracy of BG meters to ensure that its accuracy is accepted by standardized guidelines.

## 1. Introduction

Diabetes mellitus (DM) is unanimously recognised as one of the principal healthcare epidemics of the 21st century [1–4]. Such remarks stem from epidemiological data highlighting the rising burden of DM as shown by the prevalence of DM increasing from 285 million to 382 million between the years 2011 and 2013 [3, 5, 6]. Although such figures are themselves alarming, what is even more disconcerting is that this inexorable increase will culminate with DM representing the 7th leading cause of mortality by the year 2030 [7]. Realising the gravity of the situation, augmented by the lack of an existing definitive treatment, healthcare systems have invested heavily in measures to dampen the ramifications of the diabetes epidemic; for the sixth consecutive year, diabetes medications accounted for the highest net ingredient cost on the NHS prescription budget [8]. Although the principle areas of expenditure are predominantly in the management of diabetic complications and diabetic medications, another area with significant investment is in glucose monitoring systems that aid in the self-monitoring of blood glucose (SMBG) [9, 10].

RETRACTED

Widely recognised as an integral component in the management of DM, numerous studies have shown that SMBG provides an effective means of controlling blood glucose (BG) levels [11–14]. By providing instantaneous feedback to the user, in the form of their current BG level, patients can achieve effective glycaemic control whilst ensuring rapid identification of BG levels that require immediate emergency intervention [15]. Moreover, rigorous control of BG levels has demonstrated a significant reduction in the development of debilitating complications which are known to reduce the quality of life [16, 17]. Reflecting the necessity of SMBG, various organisations such as the National Institute of Health and Clinical Excellence (NICE) and the American Diabetes Association (ADA) regard the SMBG as an integral feature in the management of DM [18, 19].

As a result of the widespread integration of SMBG in healthcare policies, the use of blood glucose monitoring systems has now become commonplace. With continuing advances in the technology underpinning such devices, the provision of BG monitors has spurred a lucrative market with fierce competition between rival manufacturers. However, with numerous devices now being available, each of the differing costs and claiming to be equal to or superior to their counterpart, there has been a continuing demand for regulation of BG meters to ensure that they conform to the same standards.

In order to do so, a network of national standards bodies, known as the International Organisation for Standardisation (ISO), have devised a series of criteria which all present and future BG monitors used in the SMBG must adhere to. Known as the “performance requirements,” the ISO has deemed the accuracy of the BG monitor paramount to its use as it is deemed imperative in correctly determining whether a patient requires any immediate intervention in their diabetes control. The ISO's most recent standards, as denoted in the German Institute for Standardisation (DIN) European Nations (EN) ISO 15197:2013, provide a refinement of the performance requirements defined in the ISO 15197:2003 guidelines (ISO 15197:2003, 2003; ISO 15197:2013, 2013). In the latter, the ISO stated that ≥95% of measurements obtained from BG monitors used for SMBG must be within ±15 mg/dL (0.83 mmol/L) of the results obtained from the manufacturer's reference method at glucose concentrations <75 mg/dL (4.2 mmol/L) and within ±20% of the laboratory reference method for glucose concentrations ≥75 mg/dL (4.2 mmol/L) (ISO 15197:2003, 2003). However, in the DIN EN ISO 15197:2013, BG monitors used in the SMBG must comply with an increased, stricter degree of accuracy. In these guidelines, ≥95% of measurements obtained from BG monitors must reside within ±15 mg/dL (0.83 mmol/L) of the results obtained from the manufacturer's reference method at glucose concentrations <100 mg/dL (5.55 mmol/L), previously 75 mg/dL (4.2 mmol/L), and within ±15% of the laboratory reference method for glucose concentrations ≥100 mg/dL (5.55 mmol/L) (the upper percentage limit previously being ±20%). Furthermore, in contrast to the previous guidelines, the new standards also stipulate the inclusion of the Parkes (Consensus) error grid, a tool utilised for determining the clinical significance of the accuracy of the BG meter [20, 21].

RETRACTED

Regarded as the international standard, manufacturers of BG monitors for SMBG must provide documentation highlighting conformity to these ISO guidelines in order to obtain the Conformitè Européenne (CE) mark required for distribution of their products within the European Economic Area (EEA). Nevertheless, previously conducted evaluation studies have shown that several manufacturers have displayed the CE mark yet have not met such accuracy requirements [22, 23]. Furthermore, whether such BG monitors comply with the newly ISO 15197:2013 criteria remains of topical interest and is yet to be established as existing literature has only been able to utilise a draft version and not the final protocol.

The principle aim of this study was to determine the quality standard of the GlucoRx Nexus Voice TD-4280 BG monitoring system. Belonging to the GlucoRx Nexus series of BG monitors, the TD-4280 has recently been commissioned for possible use in the outpatient setting in the SMBG of diabetic patients under the care of our department. Claiming to conform to the ISO 15197:2003 guidelines, as identified by the CE mark, the TD-4280 offers a less expensive option than its present alternatives. Although studies have been conducted on determining the system accuracy of several BG monitors, no such literature exists for this specific model. In light of this lack of data, we devised a study to (1) determine whether the TD-4280 adhered to the ISO 15197:2003 accuracy guidelines and (2) identify if the accuracy of the TD-4280 complied with the newly released ISO 15197:2013 standards.

## 2. Study Design and Methods

This study was registered and approved as an audit at the Countess of Chester Hospital NHS Foundation Trust (CoCH), Cheshire, United Kingdom. As the variables investigated in this study were included in the audit protocol, it negated the necessity of both ethical approval and patient consent; however all areas of the investigation were conducted within an ethical framework.

RETRACTED

### 2.1. Subject Selection and Test Protocol

105 adult patients (≥18 years of age) with either DM or normal glucose metabolism were included in this study on the basis of being referred by their primary care physician for laboratory analysis of their venous blood glucose. Following withdrawal of venous blood at the antecubital fossa by a trained phlebotomist, clinical personnel involved in conducting the study drew a small quantity of blood from the sample using a disposable pipette and, in accordance with the manufacturer's guidelines, placed this onto the test strip and recorded the blood glucose concentration displayed on the BG meter in mmol/litre. Following this, the initial sample of blood obtained from the patient was then sent for determination of the plasma blood glucose using the reference measurement (see below). Results from this method were then accessed on the secure data management software MEDITECH, wherein both plasma blood glucose readings obtained from the reference measurement (in mmol/litre) and patient characteristics were recorded.

### 2.2. Self-Monitoring of Blood Glucose System

In our study, the only SMBG system under investigation was the GlucoRx Nexus Voice TD-4280 BG meter manufactured by TaiDoc Technology Corporation, Taiwan, and its corresponding test strips, the GlucoRx Nexus family Blood Glucose Test Strips, which determines the BG concentration through the glucose oxidase (GOx) method. To ensure the functionality of the BG meter, quality control measures were performed on a daily basis using the GlucoRx approved TaiDoc Control Solution (lot number: WA12K002; expiry date: 11/2014) prior to the test procedure. Throughout the study, each test was performed by clinical personnel who had familiarised themselves in how to operate the BG meter, the limitations of said device, both the safety and test protocol, and how to obtain the relevant data required for this study from the device. Furthermore, each test was performed within the confines of a laboratory setting which had its temperature and humidity controlled to the operating ranges denoted in the manufacturer's protocol (2–32°C; <85% relative humidity).

### 2.3. Reference Measurement

Reference measurements were determined on site at the CoCH using the UniCel DxC 800 SYNCHRON Clinical System (Beckman Coulter, High Wycombe, United Kingdom) which determines the plasma glucose concentration of blood samples using the glucose oxidase (GOx) method. In order to verify the measurements reported by the UniCel DxC 800 SYNCHRON Clinical System, the accuracy was verified following calibration with SYNCHRON Systems AQUA CAL 1 and 2 (Beckman Coulter, High Wycombe, United Kingdom), in addition to internal and external quality control measures being conducted as required by the CoCH.

RETRACTED

### 2.4. Statistical Analyses

Statistical analyses of the entire data set were conducted at the CoCH. Data was excluded from statistical analyses if reference measurements were absent; an incomplete data set had been recorded or either a technical error or a handling error had occurred during the processing of the blood glucose samples. Following such exclusion criteria, 105 complete data sets were available for statistical analyses. All statistical analyses were performed using the statistical software GraphPad Prism 6 and Microsoft Excel with BG concentrations being converted from mmol/L to mg/dL by multiplying each value by a factor of 18.0182. All converted BG concentrations were quoted to 2 decimal places and the subsequent accuracy percentages calculated quoted to 3 significant figures.

In order to determine whether the accuracy of the BG device conformed to the standards established by the DIN EN ISO 15197:2003 (ISO 15197:2003, 2003), calculations were initially done to determine the relative number of BG concentrations recorded from the GlucoRx TD-4280 device that were within ±15 mg/dL (0.83 mmol/L), ±10 mg/dL (0.55 mmol/L), and ±5 mg/dL (0.28 mmol/L) of the BG concentrations obtained from the reference measurement at BG concentrations <75 mg/dL (4.2 mmol/L). Moreover, calculations were also conducted to determine the number of BG concentrations recorded from the GlucoRx TD-4280 BG meter that were within ±20%, ±15%, ±10%, and ±5% of the BG concentrations obtained from the reference measurement when the BG concentration was ≥75 mg/dL (4.2 mmol/L). To evaluate whether the BG meter overall satisfied the accuracy criteria specified in the DIN EN ISO 15197:2003, the number of results obtained from the BG meter within ±15 mg/dL (0.83 mmol/L) of the reference measurement at BG concentrations <75 mg/dL (4.2 mmol/L) was added to the number of results obtained from the BG meter that were within ±20% of the reference measurement at BG concentrations ≥75 mg/dL (4.2 mmol/L). This was then converted to a percentage relative to the total number of readings (*n* = 105) and the meter was deemed compliant with the accuracy requirements if it matched the ≥95% criterion specified by the DIN EN ISO 15197:2003.

In addition to determining whether the GlucoRx TD-4280 adhered to the accuracy requirements stipulated in the DIN EN ISO 15197:2003, calculations were also done to identify whether the accuracy of the BG meter was in concordance with those defined in the DIN EN ISO 15197:2013 (ISO 15197:2013, 2013). This was achieved in a similar manner to the above but in this instance the number of BG concentrations recorded from the BG meter was within ±15 mg/dL (0.83 mmol/L), ±10 mg/dL (0.55 mmol/L), and ±5 mg/dL (0.28 mmol/L) of the BG concentrations obtained from the reference measurement for BG concentration <100 mg/dL (5.55 mmol/L; was previously 4.2 mmol/L). Furthermore, calculations were done to determine the number of BG meter readings within 15% (previous upper limit being 20%), ±10%, and ±5% of the reference measurement at BG concentrations ≥100 mg/dL (5.55 mmol/L). To determine whether the BG meter adhered to the accuracy requirements of the newer ISO 15197:2013 protocol, the relative number of results recorded from the BG meter that were within ±15 mg/dL (0.83 mmol/L) of the reference measurement at BG concentrations <100 mg/dL (5.55 mmol/L) was added to the relative number of results recorded from the BG meter that were within ±15% of the reference measurement at BG concentrations ≥100 mg/dL (5.55 mmol/L). This figure was then converted to a percentage relative to the total number of complete data sets available for analysis (*n* = 105) and the BG meter was deemed accurate within the new guidelines if the percentage matched the ≥95% accuracy requirements stipulated in the DIN EN ISO 15197:2013 guidelines.

RETRACTED

In order to provide a visualisation of the overall accuracy of the GlucoRx TD-4280 BG meter, Bland-Altman plots, otherwise known as difference plots, were constructed to illustrate the deviation of measurements obtained from the BG meter relative to the values recorded from the reference measurement. By plotting the difference in BG measurements recorded between both methods (glucose value from the BG meter subtracted from the glucose value recorded by the reference laboratory method) against the mean BG concentration for each sample (glucose value from the BG meter added to the glucose value from the laboratory method and then divided by two), we subsequently determined the degree of agreement between both techniques in the form of the average bias. Using the Bland-Altman formula [24], the average bias and its associated 95% limits of agreement (LoA), which equates to approximately 1.96 multiplied by the standard deviation, delineate the overall measuring error of the GlucoRx TD-4280 BG meter; this value incorporates the presence of both random errors and any systematic deviations between the different measurement methods used. In addition to this, a further Bland-Altman plot was also constructed to illustrate the degree of agreement between the measurements obtained from the GlucoRx TD-4280 relative to the accuracy standards required in both the DIN EN ISO 15197:2003 and the ISO 15197:2013 guidelines (ISO 15197:2003, 2003; ISO 15197:2013, 2013).

RETRACTED

As stated in the DIN EN ISO 15197:2013 guidelines (ISO 15197:2013, 2013), the clinical significance resulting from any inaccurate measurements made by the GlucoRx TD-4280 BG meter was determined using the Parkes (Consensus) error grid [20]. Consisting of five zones labelled A to E, each of differing clinical outcomes (Table 1), the predefined lines demarcating the boundaries of each region within the grid were plotted using the coordinates established by Pfützner et al. [25]. Each data set recorded from our study was then incorporated within the graph and the number of points within each region was then expressed as a percentage of the total number of samples. Any resulting bias between measurements obtained from both methods was deemed clinically insignificant if the number of results within regions A and B was ≥99%, a requirement all BG meters must adhere to in order to meet the latest ISO 15197:2013 guidelines and be awarded the CE mark.

## 3. Results

### 3.1. Patient Characteristics

With an average age of 63 years (range of 18 to 97 years), samples from 57 men and 48 women were tested over the course of the study and had their blood glucose analysed by both the BG meter and the reference method. Of the 105 individuals from whom blood samples were obtained, 22 had an underlying diagnosis of T2DM, 5 had a diagnosis of T1DM, and the remaining cohort had no underlying abnormalities with their glucose metabolism.

### 3.2. System Accuracy Evaluation

The overall accuracy of the GlucoRx Nexus TD-4280 BG monitoring device relative to both the DIN EN ISO 15197:2003 and 15197:2013 guidelines is shown in Tables 2 and 3. Moreover, Table 3 provides the percentage of recordings obtained from the GlucoRx Nexus TD-4280 BG meter that were within the accuracy limits set by each particular guideline. As stated by both versions of the ISO guidelines, ≥95% of the measurements recorded from the BG meter must be within the accuracy limits stipulated by that version of accuracy guidelines. However, as highlighted by the results in Table 3, only 92.4% of the readings from the GlucoRx Nexus TD-4280 BG meter were within the accuracy limits outlined in the ISO 15197:2003 protocol, thereby meaning it does not comply with the minimum accuracy requirements stated in that document. Similarly, with regard to the latest 15197:2013 criteria, the GlucoRx Nexus TD-4280 once again fails to achieve the minimum accuracy criteria as only 86.7% of readings were within the acceptable accuracy limits. Furthermore, as shown by Table 2, the number of BG recordings recorded by the BG meter within the stated BG concentration categories decreases as the margin of difference between the BG meter and the reference laboratory method becomes narrower. Subsequently, the accuracy of the GlucoRx Nexus TD-4280 not only fails to adhere to requirements in both versions of the ISO guidelines but, additionally, shows greater discrepancy in the BG values compared to the reference laboratory method when there is a smaller margin of difference in the BG concentration categories.

RETRACTED

In addition to this, Figure 1 provides an illustration of the results obtained from Table 3, whereby the agreement between the measurements obtained from the GlucoRx Nexus TD-4280 and the reference method relative to the ISO guidelines is provided. From the figure, 8 measurements were noted as not conforming to the accuracy limits set by the 15197:2003 protocol (indicated as the green points), thereby indicating that the remaining 97 samples (92.4%) were within limits. Similarly, Figure 2 identifies that 14 readings were not within the accuracy limits set in the 15197:2013 guidelines (indicated by both the green and blue points); thus 91 measurements (86.7%) were within the accuracy limits.

The bias of the measurements obtained from the GlucoRx Nexus TD-4280 BG meter relative to the reference method is shown in Figure 2. As illustrated by Figure 2, the average bias of the GlucoRx Nexus TD-4280 was 11.45 ± 25.77 mg/dL (0.64 ± 1.43 mmol/L) which equates to a percentage of 7.1% ± 14.91%. Clinically, such bias has little impact on BG measurements obtained provided they are not near the extremes of the clinically accepted range (70 to 130 mg/dL; 4 to 7 mmol/L). Nevertheless, if this does occur, then the bias associated with the BG meter may subsequently lead to an overestimation or an underestimation of the real BG concentration, potentially leading patients to receive unwarranted treatment or not receive necessary treatment. However, the Parkes error grid shown in Figure 3 highlights that, regardless of the bias associated with the GlucoRx Nexus TD-4280 leading to a possible over- or underestimation of the BG concentration, the effects of this on the patient, with regard to their clinical outcome, would be clinically insignificant. This is attributed to the fact that 98.1% of readings (*n* = 103) were within region A (points in red) and 1.9% (*n* = 2) of measurements were within zone B (points in green) for BG meter-derived BG readings of 185.6 mg/dL (10.3 mmol/L) and 192.8 mg/dL (10.7 mmol/L) which when compared to the BG results obtained from the reference method equated to a BG value of 149.6 mgd/dL (8.3 mmol/L) and 136.9 mg/dL (7.6 mmol/L), respectively. Both of these regions are the clinically safe regions. Furthermore, the GlucoRx Nexus TD-4280 exceeded the ISO 15197:2013 guideline requirement, whereby ±99% of all measurements from the meter, compared to those obtained from the reference method, should reside within zones A and B as 100% of all readings were within these two regions.

RETRACTED

## 4. Discussion

The aim of this study was to determine whether the accuracy of the GlucoRx Nexus TD-4280 BG monitoring device complied with the accuracy requirements outlined in both the DIN EN ISO 15197:2003 and 15197:2013 guidelines. Following our investigation, we identified that the BG meter failed to adhere to the minimum accuracy requirements stated in the ISO 15197:2003 guidelines, despite the manufacturer claiming otherwise and the BG meter being awarded the CE mark. Although we are believed to be the first to specifically evaluate the accuracy of the GlucoRx Nexus TD-4280 BG meter, other pieces of literature have conducted similar accuracy evaluation studies on a plethora of other BG meters presently marketed for the SMBG. Although the majority have been identified as conforming to the ISO guidelines [26–29], other studies have identified findings similar to ours. One such study, by Freckmann et al. [22], identified that 11 out of 27 BG meters for the SMBG failed to meet the accuracy limits set by the ISO 15197:2003 guidelines in spite of the fact that specific BG meter obtains the CE mark. Similarly, another study also conducted by Freckmann et al. [23] revealed the same predicament, whereby 7 out of 34 BG meters which had not been tested previously failed to adhere to the minimum accuracy performance requirements in the ISO 15197:2003 yet once again were noted to be CE certified.

In contrast to the ISO 15197:2003 guidelines, the ISO 15197:2013 protocol defines a narrower, more stringent accuracy performance requirement over its predecessor. Such alterations have been devised to principally ensure a greater degree of accuracy from the measurements obtained from the BG meter at hand, thereby allowing patients to have a greater ability to thoroughly control their diabetes whilst concurrently ensuring that emergency situations relating to hyperglycaemia or hypoglycaemia are correctly identified and treated. Nevertheless, our study shows that, in addition to the GlucoRx Nexus TD-4280 BG meter failing to meet the ISO 15197:2003 accuracy criteria, it also fails to conform to the minimum accuracy performance requirements outlined in the latest ISO 15197:2013 guidelines. Although we are the first to document such a finding for the GlucoRx Nexus TD-4280 BG monitoring system, previous studies have noted a similar lack of accuracy compliance to the latest guidelines, albeit using a draft version of the ISO 15197:2013 guidelines and not the full protocol released in June 2013 [23].

RETRACTED

Over the course of the study, several limitations were encountered with the first relating to the reference guidelines used to determine the accuracy of the BG meter. Although the performance requirements apply to the full range of clinically significant BG concentrations, the accuracy of the BG meter may exhibit varying measurement accuracies across this spectrum. In fact, such issues have been raised in previous literature, whereby discussions have been raised as to the notion of determining the accuracy of BG meters in the context of clinically important BG concentrations ranging from BG levels specifically representing hypoglycaemia to BG values representing hyperglycaemia [30, 31]. By doing so, it may provide the basis of differentiating the accuracy of the BG meter relative to different clinical scenarios, thereby increasing the likelihood of delivering the appropriate clinical intervention for each patient. Another area of limitation during this study related to the protocol used to conduct the study. In addition to the lack of repeatability of measurements, the measurement error inherently attributable to the reference method used may potentially reduce the reliability of the results. Furthermore, as varying haematocrit levels are known to affect the BG measurements, it would have been beneficial to identify whether there was any bias in the measurements obtained from the GlucoRx Nexus TD-4280 BG meter relative to the haematocrit level across the range of our samples [32].

Alongside our study being able to determine whether the GlucoRx Nexus TD-4280 meets the accuracy requirements stated in the ISO guidelines, we were able to delineate the clinical consequences resulting from possible inaccurate measurements. By illustrating the mean bias (mean difference) between the BG concentrations obtained from the GlucoRx Nexus TD-4280 and the reference method (Figure 2), in addition to the Parkes error grid identifying the various zones of differing clinical outcomes (Figure 3), we have identified that whilst not necessarily being accurate, the difference in results obtained from the GlucoRx Nexus TD-4280 compared to the reference method caused little to no effect on the treatment required by the patient; only two of the points resided in region B (correspond to BG readings from the BG meter of 185.6 mg/dL (reference laboratory BG reading: 149.6 mg/dL) and 192.8 mg/dL (reference laboratory BG reading: 136.9 mg/dL)). Such findings contrast existing literature, whereby the inaccuracies inherent to BG meters failing to comply with ISO guidelines place patients at significant risk of incorrect clinical interventions [22, 23].

RETRACTED

With healthcare systems such as the NHS presently struggling to cope with the economic recession, augmented by the costs associated with the management of DM, organisations are now selecting the options that retain a degree of acceptable quality yet are the most cost-effective. In light of this, one would naturally be inclined to select the most cost-effective BG meter as such meters, if they are available for purchase on the market, must presumably adhere to the minimum accuracy requirements outlined by the ISO to obtain the CE mark. However, we have demonstrated that this is not necessarily the case as, despite being awarded the CE mark, our accuracy evaluation study showed that the GlucoRx Nexus TD-4280 BG monitoring device fails to adhere to both the ISO 15197:2003 and the ISO 15197:2013 accuracy requirements. Although there are several possible reasons for this meter being inaccurate [33], BG meters should not be deemed accurate simply due to the CE mark as the acquisition of the most cost-effective BG meter, in the absence of an internal evaluation of the accuracy performance, may place patients at risk of receiving unnecessary treatment or not receiving potentially lifesaving interventions due to inaccurate measurements.

## 5. Conclusion

Despite attaining the CE mark, our study showed that the GlucoRx Nexus TD-4280 BG meter used for the SMBG failed to comply with the accuracy requirements of both the DIN EN ISO 15197:2003 and 15197:2013 guidelines. Although the clinical ramifications of such inaccurate measurements were deemed minute, inaccurate meters have the inherent risk of either overestimating or underestimating the patient's BG concentration, thereby placing patients at risk of either receiving unnecessary treatments or not receiving potentially life-saving therapeutic interventions. Therefore, our study demonstrates the importance of internally validating the accuracy of BG meters to ensure that the accuracy of such meters is within the accepted standardised guidelines.

## Figures and Tables

**Figure 1:** Bland-Altman plot demonstrating the overall system accuracy of the blood glucose measurements obtained from the GlucoRx Nexus TD-4280 compared to accuracy requirements stated in both the DIN EN ISO 15197:2003 (solid line) and 15197:2013 guidelines (dashed line). Blood glucose recordings outside the constraints of these lines are outside the accuracy limits accepted by that specific guideline protocol (green = outside accuracy requirements stated in DIN EN ISO 15197:2003; *n* = 8) (green + blue = points outside the accuracy limits defined in 15197:2013; *n* = 14).

RETRACTED

**Figure 2:** Bland-Altman plot demonstrating the relative bias of the blood glucose measurements and its associated 95% limits of agreement, obtained from the GlucoRx Nexus TD-4280 compared to those recorded from the reference measurement (SD; standard deviation).

**Figure 3:** Parkes (Consensus) error grid analysis demonstrating the clinical significance of the results obtained from the GlucoRx Nexus TD-4280. Each region demarcates a zone where a measurement would lead to differing clinical outcomes. Points outlined in red indicate measurements within zone A (*n* = 103) and points outlined in green indicate blood glucose measurements that fell within zone B (*n* = 2).

**Table 1:** Overview of the clinical significance resulting from inaccurate measurements within each region of the Parkes (Consensus) error grid.

Region	Clinical significance
A	Measurements are clinically accurate and have no effect on the clinical action required
B	Measurements lead to an altered clinical action but have little to no effect on the clinical outcome
C	Measurements lead to an altered clinical action which will affect the clinical outcome
D	Measurements lead to an altered clinical action which could be of significant medical risk
E	Measurements lead to an altered clinical action which could have dangerous consequences

**(a):** 

	DIN EN ISO 15197:2003						
	Blood glucose concentration <75 mg/dL (<4.2 mmol/L) (*n* = 5)			Blood glucose concentration ≥75 mg/dL (≥4.2 mmol/L) (*n* = 100)			
Blood glucose concentration categories defined in guidelines	±5 mg/dL (0.28 mmol/L)	±10 mg/dL (0.55 mmol/L)	**±15 mg/dL** **(0.83 mmol/L)**	±5%	±10%	±15%	**±20%**
Number of results within category	1/5	2/5	**4/5 **	38/100	77/100	87/100	**93/100 **
Percentage of results within category (%)	20	40	**80**	38	77	87	**93**

**(b):** 

	DIN EN ISO 15197:2013					
	Blood glucose concentration <100 mg/dL (<5.55 mmol/L) (*n* = 34)			Blood glucose concentration ≥100 mg/dL (≥5.55 mmol/L) (n = 71)		
Blood glucose concentration categories defined in guidelines	±5 mg/dL (0.28 mmol/L)	±10 mg/dL (0.55 mmol/L)	**±15 mg/dL** **(0.83 mmol/L)**	±5%	±10%	±15%
Number of results within category	22/34	26/34	**31/34**	26/71	59/71	**60/71**
Percentage of results within category (%)	64.7	76.5	**91.2**	36.6	83.1	**84.5**

**Table 3:** Overall determination of the accuracy of the GlucoRx Nexus TD-4280 blood glucose monitoring device relative to the accuracy limits defined in both the ISO 15197:2003 and ISO 15197:2013 guidelines.

	DIN EN ISO 15197:2003	DIN EN ISO 15197:2013
Accuracy limits set by guideline	±15 mg/dL (0.83 mmol/L) and ±20%	±15 mg/dL (0.83 mmol/L) and ±15%
Percentage of results required to be within this limit for meter to be deemed accurate	≥95%	≥95%
Number of results obtained within this limit	97/105	91/105
Percentage of results obtained within this limit (%)	**92.4**	**86.7**
Are ≥95% of the readings within the accuracy limits set in guidelines? (Yes/no)	**No**	**No**
